# A phase II trial of neoadjuvant IMRT-based chemoradiotherapy followed by one cycle of capecitabine for stage II/III rectal adenocarcinoma

**DOI:** 10.1186/1748-717X-8-130

**Published:** 2013-05-29

**Authors:** Ji Zhu, Weilie Gu, Peng Lian, Weiqi Sheng, Gang Cai, Debing Shi, Sanjun Cai, Zhen Zhang

**Affiliations:** 1 Department of Radiation Oncology, Fudan University Shanghai Cancer Center, No. 270, Dong’An Road, Shanghai 200032, China; 2 Department of Colorectal Surgery, Fudan University Shanghai Cancer Center, Shanghai 200032, China; 3 Department of Pathology, Fudan University Shanghai Cancer Center, Shanghai 200032, China; 4 Department of Oncology, Shanghai Medical College, Fudan University, Shanghai 200032, China

**Keywords:** Rectal cancer, Intensity-modulated radiation therapy, Neoadjuvant chemoradiotherapy

## Abstract

**Purpose:**

Neoadjuvant chemoradiation has become the standard treatment in locally advanced rectal cancer (LARC) and improves local control. This study explored the feasibility of an intensified chemoradiation treatment followed by one cycle of capecitabine before surgery for LARC.

**Methods and materials:**

Patients with histologically confirmed, newly diagnosed, locally advanced rectal adenocarcinoma (cT3-T4 and/or cN+) located within 12 cm of the anal verge were included in this study. Patients received intensity-modulated radiation therapy (IMRT) to the pelvis (total dose 44 Gy in 20 fractions), as well as concurrent oxaliplatin (50 mg/m^2^ d1 weekly) and capecitabine (625 mg/m^2^ b.i.d. d1–5 weekly). One cycle of capecitabine (1000 mg/m^2^ b.i.d. d1–14) was given two weeks after the completion of concomitant chemoradiation, and radical surgery was scheduled six weeks after chemoradiation.

**Results:**

Between October 2007 and November 2008, a total of 42 patients were enrolled in the study (median age 51 years; 31 male). Of these, 38 underwent surgical resection and 4 refused radical surgery because of almost complete primary tumor regression and complete symptom relief after neoadjuvant therapy. Fifteen patients underwent sphincter-sparing lower anterior resection. Six patients had a pathological complete response (pCR). The incidence of grade 3 hematologic, gastro-intestinal, and skin toxicities were 4.7%, 14.3%, and 26.2%, respectively. Grade 4 toxicity was not observed. Surgical complications (incisional infection within 2–3 weeks after surgery) were observed in 5 patients. Good responders (defined as TRG 3–4) had a significant difference in DFS (81.6% vs. 16.8%, respectively; p = 0.000) and OS (83.9% vs. 40.7%, respectively; p = 0.007) compared to those who were evaluated as TRG 1–2.

**Conclusions:**

Our study indicates that neoadjuvant chemoradiation followed by one cycle of capecitabine before surgery has a good treatment efficacy, with only mild toxicities associated with chemoradiation and acceptable surgical complications. Treatment response was an early surrogate marker and correlated to oncologic prognosis.

## Introduction

Neoadjuvant chemoradiation (CRT) followed by total mesorectal excision is the standard of care for patients with locally advanced rectal cancer (LARC). One of the benefits of neoadjuvant CRT is that patients with increased tumor downstage, such as pathological complete response (pCR), may have a better treatment outcome.

In a previous trial, patients with pathological stage T0-2 after preoperative CRT had significantly better long-term survival compared to those with less tumor downstage, such as pathological T3-4 tumors [1]. In an Italian retrospective study of 566 pCR patients, the 5-year rate of disease-free survival (DFS), overall survival (OS) and cancer-specific survival after neoadjuvant therapy increased to 85%, 90% and 94%, respectively [2]. Compared with results from other studies in stage II/III rectal cancer patients, these reports are encouraging and indicate that pCR may be considered an important potential prognostic factor in neoadjuvant CRT. Therefore, increasing the pCR rate is a key goal and neoadjuvant chemoradiotherapy may be an effective therapy for LARC patients.

In a retrospective analysis of 3,157 patients enrolled in seven randomized Phase III trials and 45 Phase II trials, the use of continuous infusion 5-FU, a second drug based on 5-FU and a higher radiation dose was associated with higher rates of pCR [3]. However, based on four reported randomized clinical trials, there was a conflict whether patients could benefit from additional oxaliplatin in the neoadjuvant CRT [4-7]. Three previous trials indicated significantly increased rates of grade 3/4 toxicity, with no improvement in pCR or sphincter preservation. However, in the CAO/ARO/AIO-04 trial, which had the largest sample size of the four trials, it was concluded that inclusion of oxaliplatin into modified fluorouracil-based combined modality treatment was feasible and led to more patients achieving a pathological complete response compared to standard treatment. Thus, a balance is needed between tumor response and toxicity in determining the optimal treatment regimen. Applied advanced radiation technology with intensified treatment may maintain this balance.

We designed this study to increase the fractional dose of radiation therapy to 2.2 Gy using an intensity-modulated radiotherapy (IMRT) technique. This approach may translate to a higher biologic effective dose (BED) compared with standard fractionation and has been proven to be effective in head and neck cancer [8,9]. Due to the uncertain toxicity in rectal cancer, the total dose used in this study was 44 Gy in 2.2 Gy/fraction, which is equivalent to 45 Gy in 1.8 Gy/fraction, assuming an α/β of 10 for tumor control [10]. Additionally, a cycle of capecitabine was scheduled two weeks after the end of chemoradiation to increase the treatment intensity without extending the interval between chemoradiation and surgery. This phase II study was approved by our institutional review board.

## Methods and materials

### Eligibility criteria

Between October 2007 and November 2008, a total of 42 patients with histologically confirmed, newly diagnosed, LARC (cT3-T4 and/or cN+) located within 12 cm of the anal verge were included in this study. Thirty-one patients were men and 11 were women, and the median age was 51 years (range, 26–73 years). All patients were ≥ 18 years of age and had a Karnofsky Performance Status score of ≥ 60, no evidence of distant metastases, adequate bone marrow function (leukocyte count > 4,000/mL and platelet count > 100,000/mL), and adequate renal and hepatic function (creatinine clearance > 50 mL/min and bilirubin ≤ 2 mg/mL). Patients were excluded if they were older than 75 years of age, had undergone previous pelvic radiotherapy or previous chemotherapy, or had previous or synchronous tumors other than nonmelanoma skin cancer. Patients suffering from the following conditions were also ineligible: ischemic heart disease, inflammatory bowel disease, malabsorption syndrome, peripheral neuropathy, or psychological disorders. Informed consent was signed and obtained from all patients before treatment.

### Pretreatment evaluation

Pretreatment evaluation was performed within two weeks before initiation of chemoradiation. The evaluation included a complete history and physical examination, including digital rectal examination, complete blood count, hepatic and renal function tests, tumor marker measurement, colonoscopy and biopsy, computed tomography (CT) of the thorax and abdomen, magnetic resonance imaging (MRI) of the pelvis, and, in selected patients, endorectal ultrasound. All patients were clinically staged with the AJCC 6th version manual.

### Combined chemoradiotherapy

#### Radiotherapy

Patients were immobilized in the prone position using a belly board and underwent a non-contrast-enhanced, planning CT scan with a 5-mm slice from the L3-L4 junction to 2 cm below the perineum. The image data sets were transferred to the PINNACLE planning system (Philips Radiation Oncology Systems, Milpitas, CA). The definitions of volumes were in accordance with the ICRU Report #83 [11]. The gross tumor volume (GTV) was defined as all known gross disease determined from CT and MRI. The clinical target volume (CTV) was defined as the GTV plus areas considered at significant risk of harboring microscopic disease, including the mesorectum (perirectal fascia), presacral region, and internal iliac lymph region. Based on our institution set-up data, the planning target volume (PTV) was generated by adding an 8-mm margin around the CTV in lateral and anterior-posterior directions, and a 10-mm margin in the superior-inferior direction. The critical normal organs at risk (OARs) outlined were the bladder, femoral heads, and small bowel. The level of outlined small bowel volume was 1 cm above the PTV.

The PTV was prescribed with a total of 44 Gy in 2.2 Gy/fraction, which was an equivalent dose to a total of 45 Gy in 1.8 Gy/fraction based on the LQ isoeffect equation [12]. The IMRT plans were generated using the inverse planning module of PINNACLE for a 6-MV linear accelerator, with five to seven coplanar fields. The D2%, D50%, and D98% were set at 41.8 Gy, 44 Gy, and 46.2 Gy, respectively. The dose of the OARs was set as low as possible and had to at least meet the following constraints: bladder, ≥ 45 Gy in 15% volume and ≥ 40 Gy in 40% volume; femoral heads, ≥ 45 Gy in 25% volume and ≥ 40 Gy in 40% volume; small bowel, ≥ 45 Gy in 65 cc volume, ≥ 40 Gy in 100 cc volume, and ≥ 35 Gy in 180 cc volume.

Patient positioning and isocenter verification were initially checked using X-ray films for anterior and lateral gantry positions by visually comparing the digitally reconstructed radiographs.

#### Concurrent and neoadjuvant chemotherapy

Capecitabine combined with oxaliplatin was administered concurrently with pelvic radiation. Capecitabine was given at a dose of 625 mg/m^2^ twice daily from Monday to Friday throughout the whole course of IMRT. Oxaliplatin at a dose of 50 mg/m^2^ was administered weekly during the four-week course of radiotherapy. Two weeks after concurrent chemoradiation, one cycle of capecitabine (1000 mg/m^2^) was administered twice daily from day 1–14 (Figure 1).

**Figure 1:** Preoperative chemoradiotherapy using capecitabine and oxaliplatin in patients with locally advanced rectal cancer.

### Surgery and histopathology

Surgery was scheduled 8 weeks after the completion of CRT. Total mesorectal excision (TME) was mandatory, whereas the form of surgery (anterior resection or abdominal-perineal resection) and whether a temporary colostomy should be performed were decided by the surgeon. All lymph nodes were examined according to standard procedures. If the number of lymph nodes was less than 12, two pathologists were needed to sign to ensure the reliability of the detection result. The circumferential rectal margin (CRM) was assessed according to the method of Quirke et al. [13], and a margin of < 1 mm was considered CRM-positive. All sections of the surgical specimens were reviewed by two pathologists. The pathologic stage (ypTN) was recorded according to the International Union Against Cancer TNM system. Tumor regression grading (TRG) was evaluated according to the criteria by Dworak et al. as follows [14]: Grade 0: no regression; Grade 1: dominant tumor mass with obvious fibrosis and/or vasculopathy; Grade 2: dominantly fibrotic changes with few tumor cells or groups (easy to find); Grade 3: very few (difficult to find microscopically) tumor cells in fibrotic tissue with or without mucous substance; Grade 4: no tumor cells, only a fibrotic mass (total regression or response).

### Adjuvant chemotherapy

All patients were recommended to receive adjuvant chemotherapy regardless of pathological stage. Adjuvant chemotherapy consisted of 6–8 cycles of Xelox with oxaliplatin (130 mg/m^2^) on day 1 and capecitabine (1000 mg/m^2^) twice daily from day 1–14, repeated every 21 days.

### Toxicity

Toxicities were evaluated and recorded weekly according to the CTC 3.0 criteria. If grade 3 toxicities occurred, the physicians determined causes and decided the response. In general, the sequence of dose reduction or suspension moved from oxaliplatin to capecitabine to radiotherapy, unless an adverse effect was strongly associated with a particular treatment.

### Endpoints and statistics

The primary endpoint for this trial was pCR rate. This study was a phase II trial of 42 patients to evaluate the treatment feasibility and efficacy of this dosing regimen. Based on the published literature, the pCR rate is approximately 10–15% for patients treated with neoadjuvant CRT. We determined that an experimental arm with a pCR rate of at least 15% would merit further study. In this study, with 42 analyzable patients, we had 80% power to reject the null hypothesis that the true number of pCR was ≤ 3, with a type I error level of 5%. Secondary endpoints included safety, sphincter preservation rate, TRG, local recurrence, DFS and OS. Sphincter preservation was defined as any procedure in which the rectal tumor was removed while leaving behind the anal sphincter.

All characteristics were described by the frequency for classified variables, by mean and standard deviations for normal distributional continuous data, and by the median for non-normal distributional continuous data.

Survival time was calculated from the beginning of CRT to the date of event or the last follow-up, and survival curves were estimated using the Kaplan-Meier method.

## Results

### Clinical characteristics

All 42 patients included in this study were diagnosed with locally advanced rectal cancer, including 28 patients with cT3 and 14 with cT4 primary tumors. Lymph node involvements were detected in 37 patients. Twenty-seven patients (64.3%) had a tumor located ≤ 5 cm from the anal verge (Table 1).

**Table 1:** Demographic and clinical features for all patients

	**n**	**%**
Gender		
Male	31	73.8%
Female	11	26.2%
Age		
≤ 50 years	20	47.6%
> 50 years	22	52.4%
Distance from anal verge		
≤ 5 cm	27	64.3%
> 5 cm	15	35.7%
cT		
T3	28	66.7%
T4	14	33.3%
cN		
N0	5	11.9%
N1	22	52.4%
N2	15	35.7%
Total	42	100.0%

### Acute oxicities and treatment compliance

All patients completed the prescribed radiation treatment to a total dose of 44 Gy in 20 fractions. The median total radiation duration was 26 days (range, 26–31 days). All patients completed concurrent oral capecitabine, and 32 patients received four cycles of weekly oxaliplatin during the course of radiotherapy. In addition, all patients received a scheduled single cycle of capacitabine two weeks after the completion of chemoradiotherapy without dose adjustment.

Most of the adverse events of this regimen were mild (grade 1 or 2). Only two patients were evaluated with grade 3 hematological toxicities, while grade 3 diarrhea and anal skin toxicities occurred in 6 and 11 patients, respectively. No grade 4 or 5 toxicities were observed (Table 2).

**Table 2:** Toxicity during the course of chemoradiation

	**Grade 1**		**Grade 2**		**Grade 3**	
	**n**	**%**	**n**	**%**	**n**	**%**
Diarrhea	15	35.71%	12	28.57%	5	11.90%
Hematologic	8	19.05%	8	19.05%	1	2.38%
Fatigue	8	19.05%	5	11.90%	3	7.14%
Radiation dermatitis	5	11.90%	18	42.86%	9	21.43%
Neurosensory	1	2.38%	1	2.38%	1	2.38%
Hand-foot syndrome	2	4.76%	0	0.00%	0	0.00%

### Surgical procedures and complications

Surgical resection was performed in 38 patients, and the median interval between chemoradiotherapy and surgery was 43 days (range, 38–53). The remaining four patients refused a radical surgery due to almost complete primary tumor regression and complete symptom relief after neoadjuvant therapy. Thirty-five patients underwent R0 surgical resection, while 15 patients underwent sphincter-sparing lower anterior resection. Incisional infection occurred in 5 patients 2–3 weeks after surgery. No other surgical complications were observed, including anastomotic fistula and abscesses.

### Pathological response and TRG score

TRG information was available in pathologic examination for all 38 patients receiving surgery. The TRG stage was Grade 4 (pCR) in 6 patients, Grade 3 in 17 patients, Grade 2 in 11 patients, and Grade 1 in 4 patients. Lymphatic/vascular invasion and neural invasion were confirmed in 4 and 8 cases, respectively. All pathological features are listed in Table 3.

**Table 3:** Surgical procedure and pathological findings

	**n**	**%**
Surgery		
Lower anterior resection	20	52.6%
Abdominal perineal resection	15	39.5%
Hartmann	3	7.9%
Lymphatic or vascular invasion		
Yes	34	89.5%
No	4	10.5%
Neural invasion		
Yes	30	78.9%
No	8	21.1%
Margin		
Negative	35	92.1%
Positive	3	7.9%
ypT		
T0	10	26.3%
T1	0	0.0%
T2	7	18.4%
T3	17	44.7%
T4	4	10.5%
ypN		
N0	22	57.9%
N1	12	31.6%
N2	4	10.5%
TRG		
4	6	15.8%
3	17	44.7%
2	11	28.9%
1	4	10.5%
Total	38	100.0%

### Follow-up and late toxicities

With a median follow-up of 26 months (range, 5–55 months), 3 patients were diagnosed with local recurrence and 10 patients were confirmed with distant metastases (5 in the liver, four in the lung, and 1 in bone). Nine patients died of rectal cancer. For the four patients that did not receive surgery, one patient died of another disease at 32 months after CRT, and the other three patients did not present any evidence of tumor failure. The 3-year local recurrence, DFS and OS rates were 12.8%, 57.4% and 66.0%, respectively (Figure 2). Late Effects on Normal Tissue / Subjective, Objective, Management and Analytic (LENT/SOMA) scales were used to evaluate late toxicities after radiation. The questionnaires were returned and available for analysis for 29/42 patients. LENT/SOMA median scores were less than 1 and no grade 3/4 late toxicities were indicated (Table 4).

**Figure 2:** Kaplan-Meier analysis of local recurrence, overall survival (OS) and disease-free survival (DFS).

**Table 4:** Late urinary, rectal, and sexual function-related toxicities on LENT/SOMA scales after neoadjuvant chemoradiation

**LENT/SOMA grade**	**Urinary function**		**Rectal function**		**Sexual function**	
	**Num**	**%**	**Num**	**%**	**Num**	**%**
0	22	75.86	26	89.66	24	82.76
1	5	17.24	2	6.90	5	17.24
2	2	6.90	1	3.45	0	0.00
3	0	0.00	0	0.00	0	0.00
4	0	0.00	0	0.00	0	0.00

*LENT/SOMA* Late Effects on Normal Tissue / Subjective, Objective, Management and Analytic.

### Subgroup analysis

The 38 patients receiving surgery were divided into two subgroups: good responders (defined as TRG 3–4) or poor responders (defined as TRG 1–2). A significant difference in DFS (81.6% vs. 16.8%, p=0.000) and OS (83.9% vs. 40.7%, p=0.007) was observed between the two groups, as shown in Figures 3 and 4, respectively.

**Figure 3:** Kaplan-Meier analysis of disease-free survival (DFS) in patients based on their response to treatment.

**Figure 4:** Kaplan-Meier analysis of overall survival (OS) in patients based on their response to treatment.

## Discussion

Neoadjuvant chemoradiation followed by surgery has been the standard care for LARC. Treatment of patients with pathologic CR after neoadjuvant chemoradiation has been shown to correlate to better local control and improved survival [1,2]. The aim of our study was to investigate the feasibility of an increased dose of chemoradiation in rectal cancer and to achieve high pCR. However, an increased dose could be accompanied by toxicities such as diarrhea. In our study, a modified strategy of neoadjuvant CRT followed by a cycle of capecitabine resulted in a pCR rate of 15.8%, which was similar to that of other reported preoperative CRT concurrent with fluorouracil and oxaliplatin (16% - 20.9%). Regarding toxicities, our study showed that the incidence of grade 3 diarrhea, hematologic toxicity, and radiation dermatitis was 11.90%, 2.38% and 21.43%, respectively. Compared with other published stage III clinical trials [4-7], the incidence of diarrhea and hematologic toxicity in our study were slight lower. However, there was a significant increase in the incidence of radiation dermatitis in our study, which might be attributed to a lower irradiation field due to a distal rectal tumor location in most cases.

IMRT is an advanced technique of high-precision radiotherapy that utilizes computer-controlled linear accelerators to deliver precise radiation doses to tumor areas. It allows higher radiation doses to be focused on regions within the tumor while minimizing the dose to surrounding normal critical structures. The data of dosimetric studies for IMRT in rectal cancer are encouraging. Henry Mok et al. compared IMRT with 3DCRT in 10 patients, and IMRT showed similar target coverage with reduced dose to the small bowel, bladder, pelvic bone and femoral heads [15]. Wolff et al. concluded that IMRT had a better conformity index and reduced the dose to the OAR compared to 3DCRT [16]. Guerrero Urbano and colleagues also reported that the volume of 45 Gy to the small bowel decreased more than 64% via IMRT [17]. By decreasing the dose delivered to normal structures, IMRT may provide a potential for increasing treatment dose to improve tumor response; however, the results of clinical outcomes for IMRT in rectal cancer are conflicting. To pursue the possibility of dose escalation, our strategy was to increase the radiation dose in two phases: the first phase increased the fractional dose to 2.2 Gy and total dose to 44 Gy, and the second phase increased the total dose based on the results from the first phase.

In the setting of neoadjuvant chemoradiation, the optimal sequencing of preoperative CRT and CT before resection of rectal cancer has been studied in several trials. In the study by Fernandez-Martos et al., four cycles of Capox were administered before preoperative CRT. They obtained a similar tumor response and a significantly decreased toxicity compared with conventional neoadjuvant CRT followed by surgery and adjuvant chemotherapy [18]. However, this treatment model prolonged the interval between initial therapy and surgery, which may increase patients’ psychological and financial burdens, especially for those with poor response to chemotherapy. Therefore, in this study, one cycle of capecitabine was prescribed in the interval between CRT and surgery, which increased the dose of preoperative therapy without delaying the schedule of surgery. Our results showed that the additional cycle of capecitabine did not increase surgical complications. Taken together, this indicates that capecitabine is effective for neoadjuvant chemoradiotherapy in patients with locally advanced rectal cancer.

Finally, our follow-up data showed that the treatment response to neoadjuvant CRT was an early indicator and correlated to long-term prognosis. Tumor response (good vs. poor) was associated with 3-year DFS (81.6% vs. 16.8%, p=0.000) and 3-year OS (83.9% vs. 40.7%, p=0.007). A similar conclusion was also reported by other studies. In a study at the MD Anderson Cancer Center, 725 patients were classified by tumor response to neoadjuvant chemoradiation (complete, intermediate and poor), and tumor response was associated with the 5-year recurrence-free survival, distant-metastasis rate and local recurrence [19]. The CAO/ARO/AIO-94 trial demonstrated that the 5-year DFS after CRT and curative resection was 86% for TRG 4 patients, 75% for grouped TRG 2+3 patients, and 63% for grouped TRG 0+1 patients (P = 0.006) [20]. In a study in Italy, 566 patients with pCR had an excellent long-term prognosis [2]. These data provide guidance with response-stratified oncologic benchmarks for different novel treatment strategies.

Based on our results, the total dose of 44 Gy in 2.2 Gy/fraction was effective and tolerable, with a pCR rate of 15.8% and mild acute toxicities. A prospective trial using a concomitant boost of 55 Gy over 25 fractions to the gross tumor is currently ongoing. In conclusion, results from our study indicate that neoadjuvant chemoradiation followed by one cycle of capecitabine before surgery has a good treatment efficacy, mild toxicities associated with chemoradiation, and acceptable surgical complications. Treatment response was an early surrogate marker and correlated to oncologic prognosis.

## Competing interest

The authors declare that they have no competing interests.

## Authors’ contributions

ZJ and GW conceived and drafted the manuscript, ZZ drafted and revised the manuscript, and all authors read and approved the final manuscript.
